# Micronutrient content in enteral nutrition formulas: comparison with the dietary reference values for healthy populations

**DOI:** 10.1186/s12937-016-0152-2

**Published:** 2016-03-31

**Authors:** Roberto Iacone, Clelia Scanzano, Lidia Santarpia, Anna D’Isanto, Franco Contaldo, Fabrizio Pasanisi

**Affiliations:** Internal Medicine and Clinical Nutrition Unit - Department of Clinical Medicine and Surgery, “Federico II” University Medical School, via S. Pansini 5, 80131 Naples, Italy

**Keywords:** Enteral nutrition, Micronutrients, Vitamins, Trace elements, Dietary reference values, Tolerable upper limit

## Abstract

**Background:**

The micronutrient content in standard enteral mixtures should be closer to the dietary reference values for a healthy population since standard enteral diets are formulated for subjects with no special nutritional needs. This study compares the micronutrient content of the most common enteral nutrition (EN) formulas with European dietary reference values (DRVs) for healthy population.

**Findings:**

Sixty-two nutritionally complete enteral formulas were considered. The micronutrient content was calculated by multiplying the value reported on the nutritional information panel of each formula by the daily dose usually prescribed. The comparison between the micronutrient content of all enteral formulas evaluated and the DRVs indicates that daily fluoride and vitamin K requirements were not covered, while an oversupply of many other micronutrients was provided. Moreover, in some enteral formulas, at a dose of 2000 Kcal/day, zinc and vitamin A content exceeded the tolerable upper limits and, for one diabetes-specific enteral formula, the chromium content exceeded the relevant European standards in both 1500 and 2000 Kcal/day diets.

**Conclusions:**

Most enteral formulas evaluated are generally suitable for patients on long-term total EN and formulas with higher content of a specific micronutrient may be a useful tool for patients affected by specific clinical conditions, at least for a period of time, then switching to standard enteral mixtures. The availability of nutritional enteral formulas, well balanced also for micronutrient intake, will further improve individualized treatments, particularly for patients on long-term total EN.

## Findings

### Introduction

Micronutrients play a key role in human nutrition by regulating several metabolic processes, and their adequate intake has a major impact on public health [1]. As the consequences of deficit or excess of micronutrient intake are known, a set of criteria has been laid down [2, 3] by an international board, defining the daily dietary reference values to guarantee an adequate healthy state and the daily tolerable upper levels to avoid possible adverse/toxic effects. Clinical conditions due to micronutrient deficiencies are not common in developed countries but inadequate micronutrient intake is often observed in malnourished patients due to an insufficient supply, malabsorption, increased losses or requirements [4]. Patients with a functional gastrointestinal tract but unable to take nutrients through the oral route receive vitamins and trace elements from daily tube-feeding formulas. In Europe, the micronutrient content in enteral formulas, as well as in foods for special medical purposes, is regulated by the directive (1999/21/EC) of 25 March 1999 [5, 6] issued by European Commission (EC). For each enteral formula, regardless of its specific composition, micronutrient content should be satisfied by supplying 1500 or 2000 Kcal/day [7].

A diet well-balanced in macro- and micronutrient content is the basis for a good health state. Most enteral nutrition (EN) formulas are designed also to meet the increased micronutrient needs in patients with increased losses or requests (e.g. moderately catabolic patients). For this reason, the micronutrient content in EN formulas is usually in excess for the needs of long term EN patients metabolically stable and without organ damage. This oversupply could be harmful in particular in patients on long-term EN. However, despite the widespread use of EN, both in hospitals and at home, studies on the micronutrient compositions in the enteral mixtures are lacking, thus an evaluation of the amount of vitamins and trace elements in the currently available products requires consideration. For these reasons, our study aims to compares the micronutrient content of 62 commercially available formulas for EN with the dietary reference values (DRVs) for the European [8] and Italian [9] populations, with the daily tolerable upper limits (UL) suggested by the European Food Safety Authority (EFSA) [3] and LARN [9], and with the relevant European standards [5, 6]. The agreement with the micronutrient DRVs and UL suggested by the European authorities [3, 8] and Italian LARN [9] is checked.

### Methods

Sixty-two nutritionally complete formulas for EN, manufactured by five different companies were evaluated. The micronutrient content was calculated by multiplying the value reported on the nutritional information panels by the daily doses of 1500 and 2000 Kcal/day. The micronutrient content was evaluated as the average content of all enteral formulas examined, by group (standard or disease-specific formulas) and by single product.

### Results

Setting DRVs at 100 % for each micronutrient and the usually prescribed daily dose of enteral formulas at 1500 and 2000 kcal/day, the average range of vitamins and trace elements contained in 62 enteral formulas compared with the DRVs is shown in Fig. 1.

**Fig. 1:** Mean percent of micronutrient content compared with DRVs. Bars (*dark gray* for 1500 Kcal/day and *light gray* for 2000 Kcal/day) indicate the mean calculated content of micronutrients in the 63 enteral formulas, compared to DRVs (fixed to 100 % as *vertical dotted line*)

Tables 1 and 2 report the DRVs, daily tolerable upper limits (UL), the limits established by the European Commission (EC Limit) and the average micronutrient content of enteral formulas grouped as standard- and disease specific at the daily doses of 1500 and 2000 Kcal/day, respectively. In assessing the average micronutrient content for the group of enteral formulas, at the doses of 1500 and 2000 Kcal/day, we found that the daily requirements for vitamin K and fluoride were not covered whereas all other micronutrients exceeded DRVs, regardless of the group of enteral formula considered. Moreover, the micronutrient content evaluated for each single enteral formula showed, in some products, a greater zinc and vitamin A content compared to the daily tolerable upper intake levels.

**Table 1:** DRVs for men and women (m/f), daily tolerable upper limits (UL), limits established by the European Commission (EC Limit) and micronutrient content (mean and range) in standard and disease-specific enteral formulas (calculated as daily intake of 1500 Kcal/day)

				Enteral formulas				
Micronutrient	DRVs m/f	UL	EC Limit Min-max	Standard *N* = 20 Mean (min-max)	Diabetes *N* = 8 Mean (min-max)	Malabsorbtion *N* = 5 Mean (min-max)	Hypercatabolism *N* = 13 Mean (min-max)	Organ Failure *N* = 16 Mean (min-max)
Trace element								
Iron. mg	10/10	-	7.5–30.0	19.1 (11.8–24.0)	17.3 (8.8–24.0)	17.0 (13.5–24.0)	18.0 (7.5–28.8)	17.8 (13.3–24.0)
Zinc. mg	11/8	25	7.5–22.5	16.8 (11.8–19.5)	17.3 (13.4–20.0)	14.5 (11.3–18.0)	20.2 (12.0–39.2)	16.3 (12.0–19.0)
Copper. mg	0.9/0.9	5	0.9–7.5	2.3 (1.5–2.7)	2.0 (1.0–2.7)	1.6 (0.1–2.7)	2.2 (0.9–3.1)	2.1 (1.3–2.7)
Iodine. mcg	150/150	600	98–525	188 (129–234)	178 (134–222)	190 (150–210)	184 (133–223)	178 (133–220)
Selenium. mcg	55/55	300	38–150	93 (62–110)	88 (66–113)	88 (75–99)	90 (54–144)	86 (63–110)
Manganese. mg	2.7/2.3	-	0.8–7.5	3.8 (1.8–5.7)	4.0 (2.2–5.3)	3.4 (2.3–5.0)	3.9 (2.7–5.7)	3.6 (1.8–5.3)
Chromium. mcg	30/20	-	19–225	111 (75–165)	161 (88–445)	80 (74–101)	95 (23–158)	106 (67–145)
Molybdenum. mcg	45/45	600	53–270	153 (61–225)	149 (122–167)	151 (113–178)	140 (54–238)	142 (67–194)
Fluoride. mg	4/3	7	0–3.0	1.7 (1.3–2.2)	1.4 (0.9–2.2)	1.5 (1.4–1.6)	1.8 (1.3–2.5)	1.6 (1.3–2.0)
Vitamin								
Vitamin A. mcg	700/600	3000	525–2700	1677 (765–2850)	1610 (854–3028)	1289 (750–1785)	1539 (750–3185)	1759 (792–2920)
Vitamin D. mcg	15/15	100	7.5–37.5	15.0 (10.0–23.2)	14.7 (10.5–25.0)	12.5 (7.5–16.8)	13.1 (9.9–23.7)	16.6 (10.0–50.0)
Vitamin E. mcg	13/12	300	7.5–45.0	22.8 (16.1–34.5)	36.0 (12.2–111.7)	19.2 (10.5–28.6)	48.4 (12.3–230.8)	34.7 (13.3–210.0)
Vitamin K. mcg	170/170	-	53–300	96 (75–129)	97 (61–150)	84 (68–99)	84 (54–115)	91 (67–115)
Vitamin C. mg	105/85	-	34–330	138 (86–165)	156 (56–278)	136 (68–210)	235 (62–646)	173 (67–840)
Vitamin B1. mg	1.2/1.1	-	0.9–7.5	2.4 (1.5–3.5)	2.2 (1.3–2.9)	2.1 (1.5–2.8)	2.1 (0.9–3.0)	2.4 (1.3–3.5)
Vitamin B2. mg	1.6/1.3	-	1.2–7.5	2.7 (2.1–4.2)	2.5 (1.7–2.9)	2.1 (1.5–2.4)	2.5 (1.7–3.9)	2.7 (1.7–4.2)
Vitamin B6. mg	1.7/1.5	25	1.2–7.5	2.8 (2.1–4.2)	2.7 (1.7–3.3)	2.4 (1.5–3.2)	2.5 (1.5–3.9)	3.0 (1.6–7.1)
Niacin. mg	18^a^/18^a^	10^b^	13.5–45.0^a^	25.9 (19.3–34.3)^a^	23.3 (14.6–30.0)^a^	27.1 (18.0–39.5)^a^	25.2 (16.0–28.9)^a^	25.3 (16.0–29.0)^a^
Folate. mcg	400/400	1000	150–750	407 (268–500)	414 (195–630)	364 (300–420)	476 (246–1950)	400 (270–500)
Vitamin B12. mcg	2.4/2.4	-	1.1–10.5	4.6 (3.1–7.1)	5.0 (4.3–7.5)	4.5 (3.0–7.9)	4.0 (2.3–5.9)	4.5 (2.7–7.1)
Pantothenic Acid. mg	5.0/5.0	-	2.3–22.5	9.4 (6.4–14.0)	8.9 (6.1–11.3)	8.0 (5.3–9.8)	8.5 (4.7–12.7)	8.6 (4.7–13.3)
Biotin. mcg	30/30	-	11–113	69 (54–75)	70 (60–87)	60 (53–75)	72 (50–104)	65 (50–75)

*N* = number of formulas considered

^a^as niacin equivalents (NE); one mg NE equals 1 mg niacin or 60 mg tryptophan, an amino acid that the liver can convert into niacin

^b^as nicotinic acid; the UL for nicotinic acid refers only to niacin from fortified food or that is in dietary supplements such as multivitamins

**Table 2:** DRVs for men and women (m/f), daily tolerable upper limits (UL), limits established by the European Commission (EC Limit) and micronutrient content (mean and range) in standard and disease-specific enteral formulas (calculated as daily intake of 2000 Kcal/day)

				Enteral formulas				
Micronutrient	DRVs m/f	UL	EC Limit Min-max	Standard *N* = 20 Mean (min-max)	Diabetes *N* = 8 Mean (min-max)	Malabsorbtion *N* = 5 Mean (min-max)	Hypercatabolism *N* = 13 Mean (min-max)	Organ Failure *N* = 16 Mean (min-max)
Trace element								
Iron. mg	10/10	-	10.0–40.0	25.4 (15.7–32.0)	23.0 (11.7–32.0)	22.6 (18.0–32.0)	24.0 (10.0–38.4)	23.7 (17.7–32.0)
Zinc. mg	11/8	25	10–30	22.4 (15.7–26.0)	23.0 (17.9–26.7)	19.3 (15.0–24.0)	27.0 (16.0–52.3)	21.7 (16.0–25.3)
Copper. mg	0.9/0.9	5	1.2–10.0	3.0 (2.0–3.6)	2.6 (1.3–3.6)	2.1 (0.2–3.6)	3.0 (1.2–4.2)	2.8 (1.7–3.6)
Iodine. mcg	150/150	600	130–700	250 (171–312)	237 (179–296)	253 (200–280)	245 (177–297)	237 (177–293)
Selenium. mcg	55/55	300	50–200	124 (82–147)	117 (88–150)	117 (100–132)	120 (73–192)	115 (84–147)
Manganese. mg	2.7/2.3	-	1.0–10.0	5.1 (2.3–7.6)	5.3 (2.9–7.0)	4.5 (3.0–6.6)	5.2 (3.6–7.6)	4.8 (2.3–7.1)
Chromium. mcg	30/20	-	25–300	148 (100–220)	215 (117–593)	106 (99–134)	127 (30–210)	141 (89–193)
Molybdenum. mcg	45/45	600	70–360	205 (81–300)	198 (163–222)	201 (150–237)	187 (73–317)	190 (89–258)
Fluoride. mg	4/3	7	0–4	2.3 (1.7–3.0)	1.8 (1.1–2.9)	2.0 (1.8–2.1)	2.4 (1.7–3.4)	2.1 (1.7–2.7)
Vitamin								
Vitamin A. mcg	700/600	3000	700–3600	2236 (1020–3800)	2146 (1138–4038)	1718 (1000–2380)	2051 (1000–4246)	2346 (1056–3893)
Vitamin D. mcg	15/15	100	10.0–50.0	20.1 (13.3–30.9)	19.6 (14.0–33.3)	16.7 (10.0–22.4)	17.5 (13.2–31.6)	22.1 (13.3–66.7)
Vitamin E. mcg	13/12	300	10.0–60.0	30.5 (21.4–46.0)	48.0 (16.2–148.9)	25.6 (14.0–38.2)	64.5 (16.4–307.7)	46.3 (17.7–280.0)
Vitamin K. mcg	170/170	-	70–400	128 (100–171)	129 (81–200)	112 (90–132)	112 (72–154)	122 (89–153)
Vitamin C. mg	105/85	-	45–440	184 (114–220)	208 (75–371)	181 (90–280)	314 (82–861)	231 (89–1120)
Vitamin B1. mg	1.2/1.1	-	1.2–10.0	3.2 (2.0–4.7)	2.9 (1.8–3.9)	2.7 (2.0–3.7)	2.8 (1.2–4.1)	3.2 (1.7–4.7)
Vitamin B2. mg	1.6/1.3	-	1.6–10.0	3.6 (2.9–5.6)	3.3 (2.3–3.9)	2.7 (2.0–3.2)	3.4 (2.2–5.3)	3.6 (2.3–5.6)
Vitamin B6. mg	1.7/1.5	25	1.6–10.0	3.7 (2.9–5.6)	3.6 (2.3–4.3)	3.2 (2.0–4.2)	3.4 (2.0–5.2)	4.1 (2.1–9.4)
Niacin. mg	18^a^/18^a^	10^b^	18.0–60.0^a^	34.5 (25.7–45.7)^a^	31.0 (19.5–40.0)^a^	36.1 (24.0–52.6)^a^	33.6 (21.3–38.6)^a^	33.7 (21.3–38.7)^a^
Folate. mcg	400/400	1000	200–1000	543 (357–667)	552 (260–840)	485 (400–560)	635 (328–2600)	534 (360–667)
Vitamin B12. mcg	2.4/2.4	-	1.4–14.0	6.1 (4.1–9.4)	6.7 (5.7–10.0)	5.9 (4.0–10.5)	5.3 (3.0–7.9)	5.9 (3.6–9.4)
Pantothenic Acid. mg	5.0/5.0	-	3.0–30.0	12.5 (8.6–18.6)	11.9 (8.1–15.0)	10.6 (7.0–13.0)	11.4 (6.3–16.9)	11.5 (6.3–17.8)
Biotin. mcg	30/30	-	15–150	92 (71–100)	93 (80–115)	80 (71–100)	95 (67–139)	87 (67–100)

*N* = number of formulas considered

^a^as niacin equivalents (NE); one mg NE equals 1 mg niacin or 60 mg tryptophan, an amino acid that the liver can convert into niacin

^b^as nicotinic acid; the UL for nicotinic acid refers only to niacin from fortified food or that is in dietary supplements such as multivitamins

Figures 2 and 3 show, respectively, zinc and vitamin A content by single enteral formula at the doses of 1500 and 2000 Kcal/day, compared to tolerable upper intake levels. With regard to zinc content, three products at 1500 Kcal/day and seven at 2000 Kcal/day exceeded daily tolerable upper level. In 13 products administered at a dose of 2000 Kcal/day, Vitamin A content exceeded the tolerable upper limit.

**Fig. 2:** Zinc content (mg) in the 63 enteral nutrition formulas evaluated. Figure shows, for each enteral formula evaluated, the calculated content of zinc at doses of 1500–2000 Kcal/day (as *dark gray bars* for 1500 Kcal/day and *light gray bars* for 2000 Kcal/day, respectively). Daily tolerable upper limit for zinc (as *vertical dotted line*) is also reported

**Fig. 3:** Vitamin A content (mcg) in the 63 enteral nutrition formulas evaluated. Figure shows, for each enteral formula evaluated, the calculated content of vitamin A at doses of 1500–2000 Kcal/day (as *bars dark gray* for 1500 Kcal/day and *light gray* for 2000 Kcal/day, respectively). Daily tolerable upper limit for vitamin A (as *vertical dotted line*) is also reported

As far as EC Limit are concerned, one enteral formula for diabetes contained a high amount of chromium (Fig. 4 and Tables 1 and 2) whilst two enteral formulas for patients with renal failure did not contain chromium. Figure 4 shows that almost all products considered had a chromium content far above DRVs.

**Fig. 4:** Chromium content (in mcg) in the 63 enteral nutrition formulas evaluated. Figures shows, for each enteral formula evaluated, the calculated content of chromium at doses of 1500–2000 Kcal/day (as *dark gray bars* for 1500 Kcal/day and *light gray bars* for 2000 Kcal/day, respectively). Dietary reference values and EC Limit at 1500 and 2000 Kcal/day (as *vertical dotted lines*) are also reported

### Discussion

Since DRVs are based on estimates of the amount of macro- and micronutrients required for healthy people, the following remarks involve mostly patients on long-term total EN in stable clinical conditions with no special nutritional needs as patients on home EN without organ failure, i.e. on exclusive lifelong enteral tube feeding. Indeed, for patients on short-term EN, the deviation from DRVs does not represent a primary concern and, for critically ill patients, the appropriate amount of micronutrients to supply is not well known and, possibly, not comparable with DRVs for healthy population. In any case, the present study is not intended to discuss the clinical effects of deficiency or excess of micronutrients in enteral formulas, as this issue has already been widely covered by various international scientific organizations and extensive reviews [2, 3, 8].

Our study confirmed that, at the calorie intake of a normal diet, micronutrients supplied in EN mixtures were often above the DRVs for healthy population [8, 9] but since the micronutrient content of most of the formulas evaluated is below the UL and within the range of the relevant European standards, it appears suitable for patients on long-term total EN. However, for some enteral mixtures, at a dose of 2000 Kcal/day, zinc and vitamin A exceeded the tolerable upper limits. As far as we know, there are no studies reporting on possible adverse effects of excessive zinc or vitamin A dosages in standard enteral formulas for patients on long-term total enteral nutrition. However, it would be more appropriate to keep the zinc and vitamin A content of standard enteral formulas at least within the limit set by the European Commission. Fluoride and vitamin K content in the evaluated enteral formulas was about 50 % lower than suggested by DRVs for healthy populations. Perhaps the fluoride and vitamin K content in enteral formulas is intentionally kept lower than DRVs, since it is believed that the daily intake of these micronutrients may also come from other sources, for example water and toothpaste for fluoride and the synthesis of menaquinones by intestinal microflora for vitamin K. When indicated and especially in the long term, supplementation could be prescribed.

Our data show that Manganese (Mn) content in enteral formulas is two folds greater than dietary reference values for healthy people, but still within the limits set by the European Commission. Mn toxicity is widely documented by the pathological absorption through inhalation and in several patients on long-term total parenteral nutrition. However, we found only one report in a patient fed enterally and with high tea consumption with potentially toxic high Mn plasma levels. On the other hand, Mn intestinal absorption is very low and finely regulated, therefore avoiding high Mn plasma levels also after a Mn rich diet. For these reasons, in our opinion the Mn content in all evaluated enteral-feeding formulas does not represent a concern.

Moreover, the upper limits indicated by the relevant European standards for both trace elements and vitamins were always observed except for chromium, which was above the upper EC Limit in one formula for diabetic patients. Since long-term excessive intake of micronutrients could be unsafe, and the daily tolerable upper limits for chromium is not known [3, 9], it is suggested to revise the chromium content at least in the enteral nutrition formulas administered for periods that exceed the limit established by European Commission.

As to the difference between the micronutrient content in enteral formulas and DRVs, several causes are possible. First, due to the heterogeneity of mixtures for EN and the wide variability in daily individual caloric/nutrient requirements, the EC directive provides the rules for vitamins and minerals allowed as relative proportions per 100 kcal: as a consequence, the daily amount of micronutrient received is related to the dose administered [5]. Secondly, in most cases and excluding fluoride and vitamin K, the low limit of range set by the EC is close to DRVs whilst the high limit is close to UL values and since manufacturers tend to keep the micronutrient content in the middle of EC range, as consequence the micronutrient content results generally higher than DRVs. Moreover, several disease-specific enteral formulas with a micronutrient adapted formulation are available for specific needs or clinical conditions, i.e., zinc-enriched enteral formulas for patients affected by burns and wound healing, formulas enriched with vitamin A to enhance immune function in cystic fibrosis, formulas with a high chromium content for diabetic patients, etc. Furthermore, for patients exclusively on EN and at high risk or with overt micronutrient deficit due to increased requirements or losses, micronutrient supplementation by enteral formulas above DRVs may be appropriate at least for a limited time, until switching to standard enteral mixtures. In any case, the 1999/21/EC directive [5] states that the limits set for some micronutrients may be exceeded in case of EN formulas for specific medical purposes and for limited periods of time and, in addition, the product labels must contain a clear warning that their use is indicated to satisfy increased nutritional requirements and that it could be unsafe for people not suffering from specific disease, disorder or medical condition.

Most patients on long term EN are in stable clinical conditions and without relevant metabolic diseases, therefore micronutrient requirements appear to be very close to those expected for the general population. Then, the micronutrient content in standard enteral formulas should be as close as possible to the DRVs for healthy populations because, as specified in the guidelines on foods for special medical purposes [10], standard diets are designed for subjects who, given their particular condition, cannot meet nutritional needs through ordinary food consumption and have no particular nutritional requirements.

In conclusion, most enteral formulas are generally suitable for patients on long-term total enteral feeding and formulas with higher content of a specific micronutrient may be a useful tool for patients affected by specific medical condition or on short-term enteral nutrition. The availability of nutritional enteral formulas, well balanced also for micronutrient intake, will further improve individualized treatment, particularly for patients on long-term total EN.

## References

[1] Shenkin A (2006). The key role of micronutrients. Clin Nutr.

[2] World Health Organization, Food and Agricultural Organization of the United Nations. Vitamin and mineral requirements in human nutrition. Second edition. 2004; 1–341. http://whqlibdoc.who.int/publications/2004/9241546123.pdf?ua=1.

[3] European Food Safety Authority (EFSA), Scientific Committee on Food, Scientific Panel on Dietetic Products, Nutrition and Allergies. Tolerable upper intake levels for vitamins and minerals. 2006; 1–478. http://www.efsa.europa.eu/it/ndatopics/docs/ndatolerableuil.pdf.

[4] Shenkin A (2008). Basics in clinical nutrition: Trace elements and vitamins in parenteral and enteral nutrition. e-SPEN, the European e-Journal of Clinical Nutrition and Metabolism.

[5] Commission Directive 1999/21/EC of 25 March 1999 on dietary foods for special medical purposes. Off. J. Eur. Communities. 1999 Apr; L91/29-L91/36. http://www.eur-lex.europa.eu/LexUriServ/LexUriServ.do?uri=OJ:L:1999:091:0029:0036:EN:PDF.

[6] European Commission. Reports of the Scientific Committee for Food (Forty-first series). Opinion on foods for special medical purposes (FSMPS). 1996 Dec; 33–40. http://ec.europa.eu/food/fs/sc/scf/reports/scf_reports_41.pdf.

[7] Iacone R, Scanzano C, Alfonsi L, Sgambati D, Fierro F, Negro G, Pastore E, D'Isanto A, Contaldo F, Pasanisi F, Santarpia L (2014). Daily macro and micronutrient supply for patients on total enteral nutrition: are they in keeping with new dietary reference intakes for the Italian population?. Nutr Metab Cardiovasc Dis.

[8] Commission of the European Communities. Reports of Scientific Committee for Food (Thirty-first series). Nutrient and energy intakes for the European Community.1993; 1–248. http://ec.europa.eu/food/fs/sc/scf/out89.pdf.

[9] Documento di sintesi per il XXXV Congresso Nazionale SINU Bologna, 22–23 ottobre 2012. LARN - Livelli di Assunzione di Riferimento di Nutrienti ed energia per la popolazione italiana. Revisione 2012. http://www.sinu.it/documenti/20121016_LARN_bologna_sintesi_prefinale.pdf.

[10] Ministero della salute. Commissione unica per la dietetica e la nutrizione. Guidelines on foods for special medical purposes (FSMP). Update December 18, 2013. http://www.salute.gov.it/imgs/c_17_paginearee_980_listafile_itemname_1_file.pdf.

